# T Tubules and Surface Membranes Provide Equally Effective Pathways of Carbonic Anhydrase-Facilitated Lactic Acid Transport in Skeletal Muscle

**DOI:** 10.1371/journal.pone.0015137

**Published:** 2010-12-13

**Authors:** Janine Hallerdei, Renate J. Scheibe, Seppo Parkkila, Abdul Waheed, William S. Sly, Gerolf Gros, Petra Wetzel, Volker Endeward

**Affiliations:** 1 Molecular and Cell Physiology, Vegetative Physiologie, Medizinische Hochschule Hannover, Hannover, Germany; 2 Abteilung Physiologische Chemie, Medizinische Hochschule Hannover, Hannover, Germany; 3 Institute of Medical Technology, Tissue Biology, University of Tampere, Tampere, Finland; 4 Department of Biochemistry and Molecular Biology, St. Louis University, St. Louis, Missouri, United States of America; Biological Research Center of the Hungarian Academy of Sciences, Hungary

## Abstract

We have studied lactic acid transport in the fast mouse extensor digitorum longus muscles (EDL) by intracellular and cell surface pH microelectrodes. The role of membrane-bound carbonic anhydrases (CA) of EDL in lactic acid transport was investigated by measuring lactate flux in muscles from wildtype, CAIV-, CAIX- and CAXIV-single ko, CAIV-CAXIV double ko and CAIV–CAIX–CAXIV-triple ko mice. This was complemented by immunocytochemical studies of the subcellular localization of CAIV, CAIX and CAXIV in mouse EDL. We find that CAXIV and CAIX single ko EDL exhibit markedly but not maximally reduced lactate fluxes, whereas triple ko and double ko EDL show maximal or near-maximal inhibition of CA-dependent lactate flux. Interpretation of the flux measurements in the light of the immunocytochemical results leads to the following conclusions. CAXIV, which is homogeneously distributed across the surface membrane of EDL fibers, facilitates lactic acid transport across this membrane. CAIX, which is associated only with T tubular membranes, facilitates lactic acid transport across the T tubule membrane. The removal of lactic acid from the lumen of T tubuli towards the interstitial space involves a CO_2_-HCO_3_^-^ diffusional shuttle that is maintained cooperatively by CAIX within the T tubule and, besides CAXIV, by the CAIV, which is strategically located at the opening of the T tubules. The data suggest that about half the CA-dependent muscular lactate flux occurs across the surface membrane, while the other half occurs across the membranes of the T tubuli.

## Introduction

Fast skeletal muscles can, during phases of maximal work – for example during a sprint -, accumulate intracellular lactic acid concentrations of up to 40–50 mM, which may be accompanied by a fall in intracellular pH to as low as 6.4 [1], [2]. At this point anaerobic glycolysis breaks down and the muscle looses its energy supply. On the other hand, slow skeletal muscles and heart muscle can take up lactic acid from the blood and use it as an important substrate for aerobic energy metabolism. Thus, the mechanisms responsible for the transport of lactic acid across the sarcolemmal membrane are decisive for the endurance of glycolytically operating skeletal muscles as well as for the extent of blood lactacidosis. Indeed, arguments have been presented to show that these mechanisms are limiting for the shuttling of lactic acid between fast muscles, erythrocytes, slow muscles and heart, respectively [2].

We have previously presented evidence from measurements of intracellular and surface pH in rat skeletal muscles showing that an extracellular membrane-bound carbonic anhydrase (CA) facilitates lactic acid transfer across the sarcolemma [3]. During lactic acid influx, for example, the presence of a CA at the extracellular surface of the muscle fiber provides a rapid source of protons by catalysing the CO_2_ hydration reaction, protons which are essential for lactate influx since the lactate-transporting monocarboxylate transporter (MCT) is a lactate-H^+^ cotransporter with a stoichiometry of 1∶1 [2]. During lactic acid efflux, the role of the extracellular CA is then to rapidly buffer the protons appearing at the membrane surface in order to avoid severe acidosis in an environment essentially lacking non-bicarbonate buffers. These functions of extracellular CA become apparent in surface pH (pH_S_) transients, alkaline during lactic acid influx and acidic during lactic acid efflux, which are small when functional CA is present and become very large when CA is inhibited. The large pH_S_ transients indicate a severe disequilibrium of the CO_2_-H^+^-HCO_3_^−^ system, which reduces lactate fluxes to about ½. The fluxes of lactic acid have been quantitated by Wetzel et al. [3] by measurements of intracellular pH (pH_i_), whose change with time during lactic acid flux can be converted to a change in intracellular lactic acid concentration by multiplication with intracellular buffer capacity. Thus, combined measurements of pH_S_ and pH_i_ with microelectrodes can be employed to assess lactate transport rates and the role of the CO_2_ hydration-dehydration reaction in this process. This experimental approach is also used in the present paper.

Our aim in the present study was a) to study which of the muscular membrane-bound CAs are involved in lactate transport and b) to assign precise functional roles to each of these CAs in the transport process. To this end, we have performed lactic acid flux measurements in fast EDL muscles of wildtype (WT), CA IV-, CA IX- and CA XIV-single, CA IV-CA XIV-double and triple knockout mice. We also have performed further subcellular localization studies of the membrane-bound CA isozymes detected in skeletal muscle, and we interpret here the flux measurements in the light of these and previous morphological results. It turns out that indeed novel specific molecular roles in sarcolemmal lactic acid transport can be attributed to each of the three isozymes. CA XIV is homogeneously distributed across the surface sarcolemma and involved in lactic acid transfer across the surface membrane. Sarcolemmal CA IX is localized only in the transverse (T) tubules and involved in lactic acid transport across the T tubular membrane. In determining this, CA IX knockout has been a unique tool allowing us to provide the first demonstration of a T tubular pathway for lactic acid. CA IV, which to a considerable part is concentrated at the T tubular openings in the surface membrane, is likely to play an important role in the diffusional transport of lactic acid out of the T tubular lumen towards the interstitial space. In the case of CA IX, the present observation represents the first physiological function that has been possible to define for this isozyme. It is interesting that it is cellular lactic acid efflux, in which CA IX is involved physiologically, since lactic acid removal is also of great importance pathophysiologically in tumors, many of which have been shown to drastically upregulate CA IX. In fact, it is well known that both MCT4 and CA IX, which we propose here to cooperate closely in eliminating lactic acid from the muscle cell via T tubules, are both up-regulated under hypoxia through HIF-1α in normal and tumour cells [4], [5].

## Results

### Membrane-bound carbonic anhydrases in mouse EDL

We have shown previously by Western Blotting that CA IV, IX and XIV are present in mouse skeletal muscle membranes, while CA XII is absent [6]. Here, we have studied the distribution the three CA isoforms in fast-twitch EDL. For that reason, single mouse EDL fibers were isolated, permeabilized with Triton X-100 and stained with primary antibodies raised against mouse CA IV, CA IX or CA XIV and fluorescently labelled secondary antibodies. We have shown previously that the antibodies against CA IV, CA IX and CA XIV are highly specific and that immunocytochemical staining is absent in muscle fibers of mice in which the CA isozyme considered had been knocked out [6], [7]. In addition, omission of the primary antibodies confirmed specificity of the CA as well as of the MCT4 and ryanodine receptor (RyR) staining. Fig. 1 shows immunocytochemical images obtained by confocal laser scanning microscopy (CLSM). In order to investigate the distribution of the three CA isozymes in the plasma membrane the microscope first was focused on the plane of the surface membrane (Fig. 1a). It is apparent that CA IV exhibits a homogeneously distributed membrane staining, but is much more concentrated at rows of dots whose pattern suggests they represent openings of T tubules. The homogeneous surface membrane staining, as well as the staining of T-tubular openings, both clearly exceed the very low background staining in CA IV-ko muscle, as it has been reported previously [6]. Using antibodies recognizing MCT4, the isoform of the lactate-H^+^ cotransporter predominantly expressed in fast muscle [8], exactly the same pattern of staining was observed. The merged images of these stainings show a perfect colocalization of CA IV and MCT4 at the T tubular openings but not on the remaining membrane surface. CA IX, although present in preparations of sarcolemmal fractions [6], is entirely absent from the sarcolemmal surface membrane (Fig. 1a), confirming a previous report [6]. CA XIV, on the other hand, shows clear homogeneous staining of the entire surface membrane and no systematic colocalization with MCT4.

**Figure 1:** Immunocytochemical CLSM images from fibers of mouse EDL muscle. a) Simultaneous exposure to antibodies against CA IV, CA IX or CA XIV and MCT4. The microscope was focussed on the plane of the fiber surface membrane. CA IV, basal homogeneous membrane staining and enrichment at entrances to T tubuli. CA IX, absence from the surface membrane. CA XIV, homogeneous surface membrane staining. b) Simultaneous staining with antibodies against CA IV, CA IX or CA XIV and RyR. The microscope was focussed on a plane inside the cell exhibiting triads. CA IV, staining of entire SR. CA IX, staining of triads (T tubules) but not SR. CA XIV, staining of light SR but not the triads (terminal cisternae of the SR and T tubules). c) Simultaneous staining with antibody against CA IX and RyR or MCT4. In the upper lane, the microscope was focussed on a plane inside the fiber free of triads; nevertheless, CA IX staining exihibits the same staining pattern as in Fig. 1b, middle lane, indicating it is associated with T tubules. In the middle lane a plane is shown, in which RyR are fully, or partially or not at all visible, causing an incomplete RyR pattern compared to that seen in Fig. 1b. Nevertheless, the staining pattern of CAIX is as complete and regular as in the lane above. This confirms that CAIX staining is associated with T tubules but not necessarily with RyR. In the lowest lane it is seen that CA IX and MCT4 are perfectly colocalized in T tubules.

In Fig. 1b single mouse EDL fibers were exposed to anti-RyR antibodies and the CLSM was focussed on a plane inside the muscle fiber. Staining of the RyR reveals a pattern typical of the arrangement of triads in skeletal muscle. With antibodies recognizing CA IV, a punctate but largely homogeneously distributed staining is obtained, suggesting staining of the entire sarcoplasmic reticulum (SR), light as well as heavy SR. This is in perfect agreement with the previously reported presence of CA IV in SR membrane fractions [9] and the earlier observation of an only partial colocalization of SR Ca^++^-ATPase (SERCA) and CA IV staining that was interpreted to indicate association of CA IV not only with terminal but also with longitudinal SR [6]. The colocalization with ryanodine receptors is highly incomplete, which is again consistent with CA IV staining of the light SR in addition to staining of the terminal SR. The minimal colocalization of ryanodine receptors and CA IV is clearly not caused by staining of T tubules, which should result in an entirely different pattern of CA IV staining, such as it is seen in the lane below for CA IX. Rather, it appears that the density of stained spots is reduced at the sites where T tubules are expected. Clearly, an increased staining intensity is not present at these sites, as would be the case if T tubules were also stained for CA IV (Fig. 1b, upper lane, left-hand picture). In accordance with this, we have observed in similar sections (unpublished) that there is also only minor overlap of intracellular CA IV and MCT4 staining. Since intracellularly only T tubules appear stained for MCT4 (see below), this confirms that the partial overlap is due to the close proximity of CA IV-stained terminal cisternae and MCT4-stained T tubules at the triads, and again argues against the presence of CA IV in T tubular membranes. In contrast to this, an example of a perfect T-tubular CA and MCT4 colocalization is shown below in Fig. 1c (lowest lane) for the case of CA IX. Fig. 1b, middle lane, shows CA IX staining in rows of high intensity dots, a pattern characteristic of T tubules, similar to what is seen for CA IV in the surface membrane, and exhibits no staining of the space in between these rows (Figs. 1b and c). The latter indicates that CA IX is not expressed in SR, which is compatible with the previous report [6] that >90% of the muscle CA IX is associated with the sarcolemmal fraction (that includes the T-tubular membranes), while the minor fraction of CA IX appearing with SR likely constitutes a contamination with T tubules rather than a genuine SR staining. The exact colocalization of CA IX with ryanodine receptors is compatible with a specific CA IX staining of T tubules that are closely attached to the triads visualized by the RyR staining. This interpretation is strongly confirmed by the data shown in Fig. 1c (see below). CA XIV in Fig. 1b (lower lane) shows punctate staining, which, as also seen in the merged image, is completely interrupted wherever triads are located. This is most easily explained by a staining of the longitudinal or light SR but not of the terminal cisternae and is compatible with the previous observation of complete colocalization of CA XIV and SERCA staining [7]. Another clear-cut implication of these pictures is the complete absence of CA XIV from T tubules. While the results presented in Figs. 1a and b largely confirm recent observations [6], [7], the following results of Fig. 1c lead to an even clearer interpretation of these data.

In Fig. 1c (upper lane), additional images have been obtained in the intracellular space of the fiber, but in a plane where triads are absent, as demonstrated by the lack of specific ryanodine receptor staining. Nevertheless, CA IX staining shows the same pattern as it does in the plane of the triads (Fig. 1b), clearly indicative of exclusive T tubular staining for CA IX. T-tubular CA IX staining is further supported by the middle lane of Fig. 1c, which shows that the pattern of CA IX staining remains complete and regular even when the intracellular plane observed exhibits an incomplete and irregular RyR pattern when compared to that seen in Fig. 1b. The association between T tubules and CA IX is further confirmed by the perfect colocalization of CA IX and MCT4 staining (Fig. 1 c, lower lane), in agreement with the findings of Bonen et al. [8].

The subcellular localization of MCT4 in mouse EDL as evident from Fig. 1 can be summarized as follows: a) there is MCT4 staining of T tubules and openings to T tubules (Fig. 1 c, lower lane, figure in the center; Fig. 1 a, all figures in the center), and b) there is surface membrane background staining between the rows of T-tubular openings (Fig. 1 a, all figures in the center). These observations verify the finding of Bonen et al. [8] of an association of MCT4 with isolated surface membranes as well as with T tubuli.

Summarizing the findings on CA localization in the sarcolemmal surface and T tubular membranes, CA IX is exclusively found in association with T tubules and is neither expressed in the surface membrane nor in the SR. CA XIV is homogeneously distributed across the sarcolemmal surface membrane, but absent in T tubuli. In contrast, CA IV exhibits some basal homogeneous staining of the surface membrane with an enriched expression at the openings of the T tubules, but is absent from the T tubules further down inside the cell.

### Lactate transport in CA IV- and CA XIV-knockout EDL muscles

Fig. 2a illustrates that lactate influx leads to an intracellular acidification, which we measure here with an intracellular pH microelectrode, and at the same time to an alkalinization on the surface of the cell, which we measure with a pH microelectrode positioned on the surface of the muscle fiber. The extracellular alkalinization occurs, because lactate influx requires the mobilization of protons, and this is strongly dependent on extracellular CA, because in the extracellular space – in contrast to the intracellular space – almost only the CO_2_-H^+^-HCO_3_^−^ system is available as a H^+^ buffer. During lactate efflux the reverse phenomena occur, with the consequence that both influx and efflux are equally dependent on CA.

**Figure 2:** Lactic acid fluxes in mouse EDL fibers. a) Schematic representation of the mechanisms of H^+^ production and H^+^ buffering associated with lactic acid influx and efflux in skeletal muscle. Fluxes can be quantitated by following the changes in intracellular pH. The changes in surface pH illustrate the associated processes of proton consumption or production on the surface membrane. b) pH_S_ and pH_I_ during exposure to and after subsequent withdrawal of lactate in the bathing solution in a WT EDL fiber. c) pH_S_ and pH_I_ during the same maneuver as in 2b in a CA IV-CA XIV double ko mouse EDL fiber. Lactate fluxes are decreased in comparison to 2b and pH_S_ transients are greatly enhanced. Note that pH_S_ curves in b and c are shifted on the pH ordinate by + 0.3 units to improve visibility. The standard bathing solution is Krebs-Henseleit solution, pH 7.4, at room temperature and equilibrated with 5% CO_2_/95%O_2_.

Figs. 2b and c show original recordings of pH_S_ and pH_i_ in mouse EDL fibers from WT animals (Fig. 2b) and from CA IV – CA XIV double knockout animals (Fig. 2c). Upon exposure of the fiber to 20 mM lactate at time 0, pH_S_ rises and pH_i_ falls as expected. The alkaline shift of pH_S_ is much more pronounced in the double ko muscle, in which all surface membrane CAs are lacking, than in WT-EDL. This increased alkaline pH shift indicates a strong limitation of H^+^ supply to the lactic acid transporter, and consequently the initial slope dpH_i_/dt is shallower in double ko than in WT muscle. The flux of lactic acid, which we define here as initial change of intracellular lactic acid concentration with time, is obtained by multiplying initial dpH_i_/dt by the total intracellular H^+^ buffer capacity. It follows therefore that lactic acid influx is reduced in double ko EDL compared to the WT muscle. In the following, we present mostly lactic acid influx values, because usually the initial slope dH_i_/dt is better defined during influx than during efflux. It should be noted that pH_i_ under normal conditions of equilibration with 5% CO_2_ is around 7.22 and identical in all knockout animals – single, double as well as triple – studied here.

Figs. 3a and b give a summary of the experimental results with CA IV and CA XIV ko mouse EDL muscle fibers. Fig. 3a shows that lactic acid influx is just below 2 mM/min in WT- EDL, is not significantly reduced in CA IV single ko EDL, but is significantly reduced in CA XIV single ko muscle. The further decrease of flux to a value below 1 mM/min seen in double ko EDL shows that lack of CA IV does have an effect on lactate transport, when CA XIV has been eliminated. Benzolamide, an extracellular CA inhibitor in muscle [3], does not further reduce lactate flux beyond that of the double ko EDL when either applied to WT fibers or to double ko fibers.

**Figure 3:** Lactate influxes and amplitudes of surface pH transients. Influxes (a) and amplitudes (b) are shown for WT fibers and for fibers lacking CA IV, CA XIV or both. On the right, both figures show the effects of the extracellular CA inhibitor benzolamide.

Fig. 3b illustrates that the changes in amplitudes of the alkaline surface pH shifts roughly correspond with the changes in fluxes. Although the pH_S_ measurement is compromised by the difficulty of positioning the electrode at a reproducible distance from the cell membrane, it is apparent that the three lowest fluxes in Fig. 3a, obtained in the absence of functional surface CAs, are associated with the three highest pH_S_ amplitudes in Fig. 3b, which is in line with the causal relation expected to exist between pH_S_ disequilibrium and flux reduction.

### Lactate transport in CA IX-knockout EDL muscles

Fig. 4a shows a comparison of the effects of CA IV, CA XIV and CA IX single ko on lactate influx in EDL fibers. It is apparent that lack of CA IX causes a marked and statistically significant reduction of flux from about 1.8 mM/min in WT to ∼1.2 mM/min, almost identical to the reduction caused by lack of CA XIV. Fig. 4b is an example showing that qualitatively identical effects are observed for lactic acid efflux, as calculated from the dpH_i_/dt seen after withdrawal of lactate from the bathing solution (Fig. 2 b, c). Both sets of data show that CA IX makes a substantial contribution to the CA-dependent lactic acid flux. Fig. 4c adds a surprising feature to this observation: while CA IX contributes significantly to flux when CA IV and CA XIV are present (two leftmost columns), it has no significant effect on flux anymore after CA IV and CA XIV have been eliminated in the double ko EDL (comparison of double and triple ko EDL in the two columns in the middle of Fig. 4c). This must be interpreted to mean that CA IX can only exert its facilitation of lactic acid flux when CA IV and CA XIV are present, i.e. the action of CA IX requires a cooperation with CA IV and CA XIV. A second information from Fig. 4c is the finding that addition of the membrane-permeable CA inhibitor ethoxzolamide to either WT or to triple ko EDL has no further effect on flux in comparison to the triple ko without inhibitor. This indicates that no other CA isoenzymes, cytosolic or membrane-bound, are involved in lactic acid transport besides CA IV, CA IX and CA XIV. The three rightmost columns in Fig. 2c indicate that the flux in WT-EDL, 1.8 mM/min, falls to ∼0.8 mM/min, when all functional CAs have been eliminated, i.e. about ½ of the total flux is dependent on CA, while the remainder does not require CA activity.

**Figure 4:** Lactate influx and efflux measurements in EDL fibers from various knockout mice. a) Lactate influxes in WT, CA IV ko, CA XIV ko and CA IX ko fibers. b) Lactate effluxes from the same combination of fibers as in 4a. c) Comparisons of lactate influxes in WT vs. CA IX ko fibers (left), in CA IV-CA XIV double ko vs. CA IV-CA IX-CA XIV triple ko (middle), and WT vs. triple ko, both in the presence of the membrane-permeable CA inhibitor ethoxzolamide (right). Columns for lactate influxes in WT, CA IV ko, CA XIV ko, and CA IV/CA XIV double ko are the same as in Fig. 3. Stars indicate significant differences from WT (* P<0.05; ** P<0.01). #(s) indicates a significant difference between the CA IX ko and the triple ko fluxes (P<0.05), &(ns) indicates that there is no significant difference between double ko and triple ko fluxes.

## Discussion

### Subcellular distribution of membrane-bound carbonic anhydrases and of MCT4

Table 1 in its first column shows previously reported activities of CA IV, CA IX and CA XIV [6]. The numbers were obtained from measurements of CA activities in preparations of sarcolemmal membrane vesicles from mouse WT, CA IV ko and CA IV-CA XIV double ko skeletal muscle. Accordingly, CA XIV is responsible for 55% of all sarcolemmal CA activity and CA IV for 30%; CA IX with 15% makes the smallest contribution. It should be noted that Western Blots of all three isozymes in WT, CA IV, CA IX and CA XIV ko mice showed no significant upregulation of any of the three CA isozymes in the ko muscles [10]. Also, the numbers given in Table 1 are compatible with those obtained by studying the CA activities of WT and CA XIV ko muscle sarcolemma [7] applying an inhibitory CA XIV antibody [11]. It follows from the immunocytochemical results described above that all sarcolemmal CA IV and CA XIV is localized in the sarcolemmal surface membrane, while all CA IX activity is associated with the T tubular membranes. This leads to the presentation of the numbers given in the 3^rd^ and 4^th^ column of Table 1.

**Table 1:** Sarcolemmal (SL) carbonic anhydrases in mouse skeletal muscle.

	CA activity of SL fraction (surface membrane +T tubuli)	CA activity of surface membranes	CA activity of T tubuli
	*U • ml/mg*	*U • ml/mg*	*U • ml/mg*
**CA IV**	1.9 (30%)	1.9* (34%)	-
**CA IX**	1.0 (15%)	-	1.0
**CA XII**	-	-	-
**CA XIV**	3.6 (55%)	3.6** (66%)	-

The activities are given in enzyme units per protein concentration in the sarcolemmal membrane fraction. They are derived from activity measurements in WT, CA IV- and CA IV-CA XIV-double-ko mouse muscle [6]. The immunoctyochemical results presented here allow us to attribute CA IV and CA XIV to the surface membrane alone and CA IX exclusively to the T tubules.

*CA IV is localized on the entire surface membrane, but greatly enriched at the openings of T tubules,

**CA XIV is homogeneously distributed over the entire surface membrane.

The subcellular distribution of MCT4 has been described by Bonen et al. [8]. Quantification of MCT4 protein in separated fractions of surface membranes, T tubuli and triads revealed similar amounts of MCT4 in surface membranes and in T tubuli, provided that the amounts associated with triads are mainly attributed also to T tubuli. This suggests that perhaps one half of the lactate transported out of fast muscles is transferred across the T tubular membranes in addition to the lactate released via the surface membranes. It seems surprising that the T tubular pathway should be efficient in comparison to the pathway across the surface membrane, and this has so far not been analysed functionally.

### Lactic acid transport across EDL surface membrane

Using the localizations of CA IV and XIV given in Table 1 and described in detail in the section Results, we can analyse the mechanism of lactic acid transport across the surface membrane in a straightforward fashion. As illustrated in Fig. 5, the MCT4 present in the surface membrane will interact with the surface carbonic anhydrases CA IV and CA XIV, which – in the absence of non-bicarbonate buffers - act to buffer the H^+^ appearing on the cell surface during efflux (as indicated in Fig. 5 by the interaction between CA XIV and MCT4) and to provide H^+^ to the transporter during lactate acid influx (as indicated in Fig. 2a, left hand side). This mechanism is suggested by the experimental finding of a reduced lactate influx in CA XIV single and CA IV-CA XIV double ko EDL (Fig. 3a) and by the increased amplitudes of surface pH transients observed in the double ko EDL (Fid. 3b). It is possible that CA XIV is more important for the surface MCT4, as both proteins are homogenously distributed across the cell surface, and CA IV may be more important for the MCT4 localized at the T tubular openings. However, since lack of CA IV alone has no significant effect on lactate flux (Fig. 3a), it appears that CA XIV, due to its presence everywhere on the surface and its contribution of 2/3 of surface CA activity (Table 1), can functionally compensate the absence of CA IV. The reverse is not true, CA IV with its more specialized localization and its contribution of only 1/3 to total surface activity, cannot compensate the lack of CA XIV as apparent from the CA XIV single ko column in Fig. 3a.

**Figure 5:** Schematic representation of the cooperation of the MCT4 and the three membrane-bound CAs in lactic acid transport across the sarcolemma. About half of lactic acid transport (in this scheme efflux) occurs via the surface membrane, supported by the buffering action of CA XIV and CA IV. The other half occurs via the T tubular membrane and is supported by the buffering action of CA IX. CA IX and half of the total sarcolemmal MCT4 are colocalized in the T tubule. The removal of lactic acid from the T tubules occurs by outward diffusion of lactate, while the H^+^ are transported out by an inward diffusion of HCO_3_^−^ in combination with an outward diffusion of CO_2_, a CO_2_- HCO_3_^−^ shuttle. This removal mechanism operates effectively in spite of the long diffusion distance from the T tubule interior to the extracellular space due to very large concentration gradients of lactate and HCO_3_^−^ that can build up along the T tubule. These gradients and the mobility of protons are much smaller in the sarcoplasm of the fiber.

### Lactic acid transport across the T tubular membrane

Due to the present finding of an exclusive localization of CA IX in T tubules, we can analyse here the mechanism of T tubular lactic acid transport. Fig. 5 illustrates our postulate that T tubular CA IX and MCT4, which microscopically are perfectly co-localized (Fig. 1c), cooperate in a fashion analogous to that of surface CA XIV and MCT4. CA IX accordingly mediates buffering of H^+^ in the T tubular lumen during lactic acid efflux and provides H^+^ to the transporter during influx. That this pathway is important, follows from the major reduction of lactate influx as well as efflux seen in the CA IX-deficient EDL (Figs. 4a, b). The marked effect is surprising in view of the small overall contribution of CA IX of only 15% to total sarcolemmal CA activity (Table 1), only half of the CA IV activity, whose knockout is of no consequence for lactate flux (Fig. 3a), and only ¼ of the CA XIV activity, whose knockout causes a loss of lactic acid flux similar to that by CA IX (Fig. 4b). This observation supports the idea that CA IX is involved in lactic acid transport in a way entirely different from CA IV and CA XIV. One question raised by the T-tubular transport mechanism is: how can lactate and H^+^ be removed efficiently from the T tubule, in which both ions have to overcome diffusion distances of up to half the muscle fiber diameter or more [12]?

In view of the "transport metabolon" consisting of MCT1 and CA II proposed by Becker and Deitmer [13], it may be asked whether the functional interactions of the membrane-bound CA isozymes are due to a physical interaction of the CA and the MCT4 molecules. In some cases this can be ruled out, namely when not even microsopic co-localization is evident as in the case of CA XIV and MCT4 (Fig. 1a), or in the case of that part of CA IV that is homogeneously distributed on the surface membrane and there shows no co-localization either. Very good co-localizations with MCT4, on the other hand, are seen in the case of the CA IV that is concentrated at the T tubular openings (Fig. 1a) and in the case of CA IX in the cross-sectioned T tubules (Fig. 1c). In these latter cases, physical interaction would be conceivable, but of course the microscopic co-localization is no proof for this.

### Lactic acid transport in the T tubular lumen

The present experimental data appear to suggest a mechanism for this process. Consideration of Fig. 4c shows that CA IX is quite effective in facilitating lactate flux as long as CA IV and CA XIV are present (two columns on the left), but after the latter two isozymes are removed, CA IX looses its effect on lactate flux (two columns in the middle). We hypothesize that this observation is related to the mechanism of lactic acid removal from the T tubule. Deeply inside the T tubule lactate concentration may become as high as it can become in the sarcoplasm, up to 40–50 mM [1], [2]. Although protons are buffered by HCO_3_^−^, pH inside the T tubule can be expected to be low, and thus we assume here for the purpose of a rough quantitative approximation that the concentration of HCO_3_^−^ deep in the T tubule is equal to the CO_2_ concentration of ∼1.3 mM (corresponding to pH 6.1) or even less. On the surface of the cell, close to the capillary, the situation will resemble more the conditions in the blood, which under conditions of exhaustive exercise in the study of Sahlin et al. [1] are characterized by a lactate concentration of ∼12 mM, a pH of 7.2, and accordingly a HCO_3_^−^ concentration of ∼16 mM. In this example, one would have concentration differences between deep inside the T tubule and the surface of the fiber of 40 to 50–12 = 28 to 38 mM for lactate, and of 1–16 = −15 mM for HCO_3_^−^. This is the situation to which the intraluminal mechanisms depicted in Fig. 5 refer to. The gradient for lactate drives lactate out of the T tubule towards the interstitium. The protons cannot diffuse as free protons because their gradient will be far too small. Mobile buffers that could mediate facilitated H^+^ diffusion [14], [15] are not present. The only known mechanism applicable in this situation is the one shown in Fig. 5: H^+^ transport out of the T tubular lumen is achieved by an inward diffusion of HCO_3_^−^ (which will partly or fully electrically compensate outward lactate diffusion) in combination with an outward diffusion of CO_2_, i.e. a CO_2_-HCO_3_^−^ shuttle for H^+^ transport. This shuttle requires that inside the T tubule HCO_3_^−^ and H^+^ react rapidly to produce CO_2_, and that at the opening of the T tubule to the interstitial space CO_2_ reacts back to produce the HCO_3_^−^, which then diffuses again down into the T tubule to supply HCO_3_^−^ for H^+^ buffering to the sites where MCT4 and CA IX are located. Thus a CA, i.e. CA IX, is needed deep in the T tubule to buffer H^+^ and produce CO_2_, and again, at the opening of the T tubule, a CA, i.e. CA IV and probably also CA XIV, is required to regenerate HCO_3_^−^. The arguments for this mechanism are: 1) it explains why CA IX can only facilitate lactic acid transport in conjunction with the surface CAs CA IV and probably CA XIV, 2) it convincingly explains the specific enrichment of CA IV at the openings of the T tubules (Fig. 1 a), a location ideally suited for this purpose as visualized in Fig. 5. Finally, two properties of CA IX make it appear especially suited for its proposed function in the T tubule. CA IX exhibits a greater tolerance towards acidic conditions in comparison to other membrane-bound CAs [16], which will allow it to remain active when pH inside the T tubule falls to much lower values than on the cell surface. Another notable property of CA IX is its resistance towards inhibition by lactate (K_I_>150 mM; [17]), which makes it especially suited for the expected high intraluminal lactate concentrations in T tubules. This situation is in contrast to the surface membrane, where much lower lactate concentrations are expected physiologically under intense exercise and where CA IV as well as CA XIV, like many other CA isoforms, have K_I_ values towards lactate in the low millimolar range ([17]; Dr. C.T. Supuran, Florence, personal communication). In concluding this section, it should be noted that the net effect of all T tubular transport mechanisms is a release of lactate and H^+^ into the interstitial space.

### Physiological significance of T tubular vs. surface membrane lactic acid transport

The relative contributions of these two pathways can be derived from the present data. Fig. 4c shows the WT level of lactate influx, ∼1.8 mM/min, and the basal CA-independent flux level, in triple ko EDL and in EDL exposed to ethoxzolamide, of 0.8 mM/min. In CA IX ko EDL, in which the CA-dependent T tubular pathway should be completely suppressed, a flux of 1.25 mM/min has been measured, suggesting that about ½ of the CA-dependent lactic acid transport occurs via the T tubule, the other half via the surface membrane. Such a distribution of the quantitative roles of flux pathways is in excellent agreement with the finding of Bonen et al. [8] of an equal allocation of the sarcolemmal MCT4 to surface membranes and T tubuli.

What may be the advantage of additionally using the T tubular pathway over only using the route through the sarcoplasm and the surface membrane? Peachey and Eisenberg [12] have shown that the T tubular system forms a close-mesh network extending all over the interior of the skeletal muscle fiber. Thus, T tubules can take up lactic acid everywhere in the cell at very short distances, and thus rapidly remove lactic acid from the sarcoplasm right where it is produced. The overall distance that has to be overcome by intracellular radial diffusion and by diffusion through the T tubule may be considered similar, and the diffusivities of lactate and HCO_3_^−^, even if considering tortuosity effects in the T tubules and in the sarcoplasm [18], are also expected to be similar. However, the volume fraction of the T system is 0.3% [19] and thus the total diffusional cross section of the T tubules will be small. In fact, there has been a long-standing speculation and discussion on whether ions are exchanged to a significant extent between the T-tubular lumen and the extracellular space [20], [21], but clear-cut evidence to our knowledge has not been obtained so far. This disadvantage of the small volume and diameter of T tubules in the present case may be overcome by the large gradients of lactate as well as HCO_3_^−^ concentration along the diffusion path through the T tubules, as explained above. These gradients are expected to be much smaller in the sarcoplasm. During acid loading of enterocytes maximal intracellular pH gradients have been measured in the order of ∼0.1 unit [22]. The intra-tubular pH gradient in the above hypothetical example would be 7.2–6.1 = 1.1 units, i.e. ten times greater than the possible intracellular pH gradient.

If we express the transport properties of sarcoplasm vs. T tubular lumen by the product D · Δc, we find that not only the concentration gradients but also the effective proton mobilities are greater within the T tubule than in the sarcoplasm. We consider here proton transport rather than lactate transport, because it is likely that in both cases proton flux constitutes the limiting step:

1) Intracellular transport of protons: D is interpreted according to the concept proposed by Junge and McLaughlin [23] as an apparent diffusion coefficient of bound together with free protons. This quantity was reported to assume a value of D_app_ = 3.8 · 10^−7^ cm^2^s^−1^ in cardiomyocytes [24], when buffering by HCO_3_^−^ is of little importance, as is the case for the low intracellular pH value considered here. Δc represents the combined intracellular concentration difference of bound and free protons, which is given by the product of intracellular pH difference, ΔpH, times the intracellular non-bicarbonate buffer capacity BF of 24 mM/ΔpH (see Methods). With an assumed ΔpH of 0.1 we obtain a proton transport rate of D_app_ · ΔpH · BF = 3.8 · 10^−7^ cm^2^ s^−1^ · 0.1 · 24 mM = 9.1 · 10^−7^ µM cm^−1^ s^−1^.

2) Intratubular transport of protons: In this case, we can approximate the H^+^ transport rate by the transport rate of bicarbonate in opposite direction, assuming that CO_2_ diffusion, due to the greater diffusivity of CO_2_ compared to HCO_3_^−^, is not rate-limiting. D · Δc is then obtained as follows. D_HCO3_- is taken to be 1.2 · 10^−5^ cm^2^ s^−1^ [25], and for Δ[HCO_3_^−^] we use the above hypothetical value of 15 mM. With this we estimate the intratubular proton transport rate to be D_HCO3-_ · Δ[HCO_3_^−^] = 1.2 · 10^−5^ cm^2^ s^−1^ · 15 mM = 1,800·10^−7^ µM cm^−1^ s^−1^.

These estimates indicate that T tubular proton transport can be ∼200 times more efficient than intracellular proton transport. This is so because a) due to the highly different pH gradients, the gradient of the molecules directly or indirectly mediating proton transport is 15/2.4 = 6.3 times greater in the T tubule than intracellularly, and b) the effective diffusion coefficient of these molecules is 32 times greater inside the T tubule than in the cytoplasm of the muscle cell. It should be noted that the intracellular pH gradients occurring while the muscle cell produces and releases lactic acid have not been measured directly and may be less than 0.1, making the intracellular proton transport pathway even less effective in comparison to the T tubular pathway. In conclusion, the small volume fraction taken up by the T tubules is counterbalanced approximately quantitatively by the properties of the proton transport inside the T tubules. This latter transport mechanism is so much more efficient than the route across the sarcoplasm that comparable contributions of both pathways to the elimination of lactic acid from the muscle cell can be expected. This constitutes a satisfactory physicochemical explanation of the experimental finding of identical sizes of lactic acid fluxes across the surface membrane and across the T tubular membrane.

It may be hypothesized in addition that during contraction T tubuli are alternatingly compressed and decompressed, thereby producing a convective flow of water and solutes along the T tubular lumina, which would further improve lactic acid transport out of the T tubuli, although at present there is no experimental evidence for such a phenomenon.

## Methods

### Ethical approval

All experiments were done according to the guidelines of the Bezirksregierung Hannover and approved by this institution (Approval ID 42500/1H).

### Animals and muscle fiber preparation

The CA IV, CA IX and CA XIV ko mice have been characterized earlier [26], [27]. They were bred on a C57BL/6J background and crossbred to obtain CA IV-CA XIV double ko and CA IV-CA IX-CA XIV triple ko animals. Mice were sacrificed by cervical dislocation and the extensor digitorum muscle (EDL) was dissected out. From the muscles, fiber bundles were prepared under a microscope as described [3].

### Electrophysiology

The membrane potential electrodes (2 MΩ), the intracellular pH microelectrode (20–30 GΩ), the surface pH microelectrode (5–10 GΩ), the latter two filled at the tip with Hydrogen Ionophore Cocktail A (Fluka), and the reference electrode were constructed as described earlier [3]. The muscle fiber bundles were subjected to moderate passive tension and placed in an open bathing chamber that was continuously perfused with Krebs-Henseleit solution equilibrated with 5%CO_2_/95%O_2_ at room temperature. One superficial single fiber of the bundle was chosen to position the intracellular pH (pH_i_) and the membrane potential electrode intracellulary and the surface pH microelectrode (pH_S_) on the cell surface. pH_i_ values in EDL fibers under control conditions were 7.22 (S.D. ±0.10, n = 23). Control pH_i_ values in muscle fibers from knockout animals and/or in the presence of benzolamide or ethoxzolamide were not significantly different from this value. pH_S_ values in control EDL fibers were on average 7.31 (S.D. ±0.09, n = 23), and again pH_S_ values of knockout fibers and fibers in the presence of CA inhibitors were not significantly different from this value. Intracellular non-bicarbonate buffer capacity was determined by exposing the muscle fibers to three different CO_2_ partial pressures: Krebs-Henseleit solution (98 mM NaCl) with 5% CO_2_, 25 mM NaHCO_3_ and 27 mM methane sulfonic acid, or with 2% CO_2_, 10 mM NaHCO_3_ and 42 mM methane sulfonic acid, or with 14% CO_2_ and 52 mM NaHCO_3_. pH_i_ was measured at these three pCO_2_ values, used to calculate intracellular [HCO_3_^−^], and Δ[HCO_3_^−^]/ΔpH_i_ yielded the intracellular non-bicarbonate buffer capacity (24 mM/ΔpH for mouse EDL, with no significant differences between wildtype and knockout muscles). For a given experimental ΔpH_i_ the bicarbonate buffer capacity was calculated applying the Henderson-Hasselbalch equation for a constant pCO_2_. The sum of both buffering factors was used to convert the initial dpH_i_/dt observed during lactate influx and efflux into lactate fluxes in mM/min. Lactate flux experiments were conducted by rapidly switching between a Krebs-Henseleit solution with 100 mM NaCl, 20 mM methane sulfonic acid (5%CO_2_) and one with 100 mM NaCl, 20 mM Na-lactate (5%CO_2_). The switch led to a decrease in pH_i_ with time, whose initial kinetics was determined as described [3]. The pHi reached a plateau during continued exposure to Na-lactate and returned gradually to the control value after the perfusion was switched back to the lactate-free solution (see Fig. 2). pH of all Krebs-Henseleit solutions employed was 7.36 at room temperature. Further details of this method to measure lactate fluxes have been reported previously [3].

### CA Inhibitors

Benzolamide (2-benzenesulfonamido-1,3,4-thiadiazole-5-sulfonamide) was a kind gift from Dr. Erik Swenson (Seattle, USA) and was used at a final concentration of 1· 10^−5^ M. Ethoxzolamide (6-ethoxy-2-benzothiazolesulfonamide) was from Sigma Aldrich (Seelze, Germany) and was used at a final concentration of 1·10^−4^ M.

### Immunocytochemistry

EDL muscle fiber bundles were fixed while subjected to passive tension with 3% paraformaldehyde and 100% methanol and permeabilized in 0.1% Triton X-100 for 5 min, and stained with primary and secondary antibodies as described [6]. Fibers were incubated with primary antibodies for 30 min. The polyclonal rabbit anti-mouse CA IV and CA XIV [11], [28], [29] and the polyclonal rabbit anti-mouse CA IX antibody (Santa Cruz Biotechnology sc-25600; Santa Cruz, CA, USA) were diluted 1∶400. Goat anti-mouse ryanodine receptor RyR (sc-8170) and goat anti-mouse MCT4 (sc-14934) antibodies were also from Santa Cruz Biotechnology and diluted 1∶200. Incubation with FITC-labelled anti-rabbit and TRITC-labelled anti-goat IgG secondary antibodies (Santa Cruz Biotechnology) was performed for additional 30 min. The subcellular localization was examined by CLSM (Leica DMIRRE, Wetzlar, Germany) and analysed with Image Span software (Leica TCS-NT).

### Statistics

The mean values of experimental results in Figs. 3 and 4 are given together with S.D. values (bars) and n ( = number of fibers investigated). Significance of differences between groups of data and WT controls were performed using One-Way ANOVA followed by Dunnett's Multiple Comparison Post Test using the program Prism 3.0. The Bonferoni Post Test for selected pairs of data groups was used to test two pairs of data groups of special functional interest (Prism 3.0).
